The article "Reduced TGF-β Expression and CD206-Positive Resident Macrophages in the Intervertebral Discs of Aged Mice" was published in 2021. Journal: Biomed Res Int.

# Reduced TGF-*β* Expression and CD206-Positive Resident Macrophages in the Intervertebral Discs of Aged Mice

**DOI:** 10.1155/2021/7988320

**Published:** 2021-07-12

**Authors:** Yuji Yokozeki, Ayumu Kawakubo, Masayuki Miyagi, Akiyoshi Kuroda, Hiroyuki Sekiguchi, Gen Inoue, Masashi Takaso, Kentaro Uchida

**Affiliations:** ^1^Department of Orthopedic Surgery, Kitasato University School of Medicine, 1-15-1 Minami-ku Kitasato, Sagamihara City, Kanagawa 252-0374, Japan; ^2^Shonan University of Medical Sciences Research Institute, Nishikubo 500, Chigasaki City, Kanagawa 253-0083, Japan

## Abstract

Age is a key factor in intervertebral disc (IVD) degeneration; however, the changes that occur in IVDs with age are not fully understood. Tissue-resident macrophages are critical for tissue homeostasis and are regulated by transforming growth factor- (TGF-) *β*. We examined changes in the proportion of resident macrophages in young versus aged mice and the role of TGF-*β* in regulating resident macrophages in IVDs. IVDs were harvested from 4-month (young) and 18-month-old (aged) C57BL/6J mice. The proportion of macrophages in IVDs was determined using flow cytometry (*n* = 5 for each time point) and the expression of *Cd11b*, *Cd206*, and *Tgfb* genes, which encode CD11b, CD206, and TGF-*β* protein, respectively, using real-time PCR. To study the role of TGF-*β* in the polarization of resident macrophages, resident macrophages isolated from IVDs from young and aged mice were treated with recombinant TGF-*β* with and without a TGF-*β* inhibitor (SB431542). Additionally, SB431542 was intraperitoneally injected into young and aged mice, and *Cd206* expression was examined using real-time PCR (*n* = 10 for each time point). The proportion of CD11b+ and CD11b+ CD206+ cells was significantly reduced in aged versus young mice, as was *Cd11b*, *Cd206*, and *Tgfb* expression. TGF-*β*/IL10 stimulation significantly increased the expression of *Cd206*, an M2 macrophage marker, in disc macrophages from both young and aged mice. Meanwhile, administration of a TGF-*β* inhibitor significantly reduced *Cd206* expression compared to vehicle control in both groups. *Conclusion*. Resident macrophages decrease with age in IVDs, which may be associated with the concomitant decrease in TGF-*β*. Our findings provide new insight into the mechanisms of age-related IVD pathology.

## 1. Introduction

Intervertebral disc (IVD) degeneration is frequently linked to low back pain [1, 2], and age is a key factor in IVD degeneration. Evidence suggests that several factors, including altered extracellular matrix components, anabolic/catabolic balance, cell senescence, and inflammation, are associated with aging-related IVD degeneration [3–6]. However, the changes that occur in IVDs with age are not fully understood.

Various kinds of macrophages, including resident macrophages and recruited macrophages, are present in degenerated IVDs [7–10]. Recruited macrophages differentiate into proinflammatory phenotype M1 macrophages, which are thought to induce inflammation in IVDs [7]. In contrast, tissue-specific macrophages, known as resident macrophages, exist in a variety of tissues [10–14]. Recent studies have demonstrated that resident macrophages exist in mouse and human IVDs [9, 10, 13]. Resident macrophages exhibit M2 phenotype and play an important role in promoting regeneration, inflammation resolution, and remodeling [15]. However, a previous study reported that resident macrophages in the heart decrease and show declining self-renewal activity with age [16]. Age-related reductions in resident macrophages in IVDs may form part of the mechanism underlying age-related IVD degeneration. However, the factors causing age-related decreases in resident macrophages remain to be determined.

Transforming growth factor-beta (TGF-*β*) signaling plays important roles in a number of cellular processes, including cell proliferation, migration, differentiation, and apoptosis, in different cell types, and is associated with aging-related pathology [17]. TGF-*β* and its receptors have been observed in nucleus pulposus and annulus fibrosus cells in young mice; the expressions of which are reduced with age [18]. Further, recent studies have reported that TGF-*β* promotes the development and homeostasis of resident macrophages in the skin and lung [19, 20]. We hypothesized that age-related decreases in TGF-*β* may alter resident macrophage populations in IVDs.

Here, we examined changes in the proportion of resident macrophages in young versus aged mice and the role of TGF-*β* in regulating resident macrophages in IVDs.

## 2. Materials and Methods

### 2.1. Animals

The study protocol received approval from the Kitasato Institutional Animal Care Committee (reference number: 2020-089). The study complied with the ARRIVE guidelines for the reporting of animal experiments. All methods were conducted based on the guidelines for the proper conduct of animal experiments by the Science Council of Japan.

Male C57BL/6J (B6) mice aged 4 (young) and 18 (aged) months (30 mice each) were housed in a housing system maintained at 25 ± 1°C and 60 ± 5% humidity with a 12 : 12-hour light : dark cycle throughout the study period.

Coccygeal (Co) 5/6, Co6/7, and Co7/8 IVDs were resected without separating the nucleus pulposus (NP) and annulus fibrosus (AF) and pooled for each measurement.

### 2.2. Flow Cytometric Analysis

IVDs were harvested from young and aged mice (*n* = 5 each) and digested with 2 mg/ml collagenase type I solution (Product no. 032-22364, Fujifilm Wako Pure Chemical Corporation, Osaka, Japan) at 37°C overnight, before being passed through a nylon mesh filter with pore size 100 *μ*m. The resulting single-cell suspensions were incubated with PE/Cy7-conjugated anti-CD45 (Clone: 30-F11, Product no. 103114, BioLegend, CA, USA) and APC-Cy7-conjugated anti-CD11b (Clone: M1/70, Product no. 101226, BioLegend) antibodies for 40 min at 4°C and subsequently treated with fixation/permeabilization solution (Product no. 420801, BioLegend). The cells were then incubated with APC-conjugated CD206 antibody (Clone: C068C2, Product no. 141708, BioLegend) for 30 min at 4°C and washed twice in wash buffer. The labeled cells were subjected to flow cytometry, in which 50,000 total events were acquired using a BD FACSVerse system (BD Biosciences, San Jose CA, USA), and the results were analyzed using FlowJo v10.7™ (Tree Star, Ashland OR, USA). Negative gates were determined using isotype control.

### 2.3. Real-Time PCR Analysis

IVDs were harvested from young and aged mice (*n* = 10 each). Standard TRIzol (Product no. 15596026, Invitrogen, Carlsbad, CA)/chloroform methods were used to extract total RNA from IVD samples. SuperScript III RT™ (Product no. 18080085, Invitrogen) was subsequently used to synthesize first-strand cDNA for use in real-time PCR with SYBR™ Green (Product no. 204054, Qiagen, Valencia CA, USA). We examined the expression of *Cd11b* (macrophage marker), *Cd206* (M2 maker), and *Tgfb* genes, which encode CD11b, CD206, and TGF-*β* protein, respectively, based on previous reports [9, 13, 21]. Primers were generated according to our previous report [9, 13, 21]. The delta-delta Ct method and the housekeeping gene *Gapdh* were used to determine relative mRNA expression levels of the genes of interest.

### 2.4. Effect of TGF-*β* Inhibitor on Resident Macrophages In Vitro

Following collagenase digestion, IVD-derived cells obtained from young and aged mice, as described above (*n* = 5), were incubated with biotin-conjugated anti-CD11b (Clone: M1/70, Product no. 101204, BioLegend) antibodies for 30 min at 4°C. After washing twice with PBS at 300 × g at 4°C, IVD cells were reacted with streptavidin-magnetic particles (Product no. 557812, BD Biosciences, San Diego, CA, USA) for 30 min at 4°C, before incubating on ice for 8 min in an IMag separation system (Product no. 552311, BD Biosciences). After aspirating the unbounded cells (CD11b-negative cells), the tube was removed from the magnetic support to obtain the CD11b-positive cells, and 5 ml of culture medium was added. The positive fraction was washed twice with culture medium (*α*-MEM with 10% fetal bovine serum) at 300 × g at 4°C, before being incubated in culture medium supplemented with 100 ng/ml recombinant mouse macrophage colony-stimulating factor (M-CSF; Product no. 576406, BioLegend) for 7 days. Following the culture period, macrophages were stimulated with culture medium (vehicle), 10 ng/ml mouse recombinant TGF-*β* (mrTGF-*β*; Product no. 7666-MB-005/CF, R&D Systems, Minneapolis, MN, USA) + 10 ng/ml mouse recombinant IL-10 (mrIL-10; Product no. 575806, BioLegend), or mrTGF-*β* +IL-10+ 1 *μ*M SB431542 (TGF-*β* inhibitor; Product no. S4317, Sigma-Aldrich, St Louis, MO, USA) for 24 hours. M2 marker (*Cd206*) expression was subsequently determined using real-time PCR analysis.

### 2.5. Effect of TGF-*β* Inhibitor on *Cd206* Expression in IVDs

Young and aged C57BL/6J mice were randomly and equally divided into control and treatment groups (*n* = 10 each). The control group received an intraperitoneal (IP) injection of 5% DMSO solution (vehicle), while the treatment group was given an IP injection of 10 mg/kg SB431542 in 5% DMSO solution. Dosage was chosen according to the optimal inhibitory effect observed at an IP dose of 10 mg/kg, as reported previously [22, 23]. After 24 hours, IVDs were harvested from young and aged mice and *Cd206* expression was determined using real-time PCR.

### 2.6. Statistical Analysis

Distribution of the data was evaluated using the Kolmogorov-Smirnov test. Mann–Whitney *U* tests were used to evaluate differences between the 4- and 18-month groups. Bonferroni multiple comparisons test with one-way ANOVA was used to determine differences among the vehicle and TGF-*β*/IL-10 or TGF-*β*/IL-10/SB431542 treatment groups.

## 3. Results

### 3.1. Proportion of Resident Macrophages and *Tgfb* Expression in Young and Aged Mice

The proportion of CD11b+ and CD11b+ CD206+ cells was significantly reduced in aged versus young mice (CD11b+, *P* < 0.047; CD11b+ CD206+, *P* = 0.009; Figure 1). Consistent with these flow cytometry findings, *Cd11b* and *Cd206* expression was also significantly reduced in aged versus young mice (*Cd11b*, *P* = 0.007; CD206, *P* < 0.001; Figures 2(a) and 2(b)). Likewise, *Tgfb* expression was significantly reduced in aged versus young mice (*P* < 0.001; Figure 2(c)).

### 3.2. Effect of TGF-*β* Inhibitor on *Cd206* Expression in Resident Macrophage Cell Culture

Expression of the M2 macrophage marker *Cd206* was significantly elevated following TGF-*β*/IL10 stimulation of macrophages derived from young and aged mice (young, *P* = 0.030; aged, *P* = 0.002; Figure 3). This increase was significantly reversed following exposure to SB431542 (young, *P* = 0.030; aged, *P* = 0.002; Figure 3). *Cd206* expression was comparable in macrophages derived from young and aged mice subjected to the same culture conditions.

### 3.3. Effect of TGF-*β* Inhibitor on *Cd206* Expression in IVDs In Vivo

An IP injection of the TGF-*β* inhibitor SB431542 significantly reduced *Cd206* expression relative to vehicle control in both young and aged mice (*P* < 0.001 and *P* = 0.047, respectively; Figure 4).

## 4. Discussion

Tissue-resident macrophages are critical for tissue homeostasis and immunomodulation. Mice lacking resident macrophages in the epidermis, known as Langerhan cells (LCs), which express IL-10 [24], develop exaggerated contact hypersensitivity. Loss of alveolar macrophages hinders the accumulation of pulmonary surfactants, ultimately causing pulmonary alveolar proteinosis [12, 25, 26]. In our study, we observed a heterogeneous population comprising CD206− and CD206+ macrophages in mouse IVDs, both of which decreased with age. Numerous studies have suggested that CD206+ resident macrophages play an important role in immunosuppression [27, 28]. In allergic skin inflammation, Th2 cytokines induce CD206+ M2 macrophage-mediated anti-inflammatory activity [28]. CD206+ M2 macrophages also show anti-inflammatory activity during endotoxemic lung injury through inhibiting the production of a number of proinflammatory cytokines [27]. The role of resident macrophages in IVDs, however, remains unclear. We hypothesized that the age-related reduction in resident macrophages may be associated with age-related IVD degeneration.

Previous studies have shown that, in addition to being self-regulatory, TGF-*β* regulates resident macrophages in adult mice [19, 20]. TGF-*β* regulates LCs, with the number of LCs shown to decrease in the absence of TGF-*β* [20]. Treatment of *R26^CreER^Tgfbr2^fl/fl^* mice with tamoxifen to delete *Tgfbr2* encoding TGF-*β* receptor 2 from all cells and tissues causes a significant decrease in alveolar macrophages [19]. In our study, *Tgfb* expression decreased with age and inhibition of TGF-*β* reduced *Cd206* expression in IVDs. Together with findings from previous studies, our results suggest that the age-related decrease in TGF-*β* leads to a reduction in resident macrophages in IVDs.

The risk of IVD degeneration is thought to be greater in aging women than men [29, 30]. A previous study showed that 17-beta-estradiol promotes TGF-*β* production in cartilaginous endplate cells derived from human IVDs [31]. Further, a recent study reported that estrogen deficiency alters the M1/M2 ratio in mouse bone marrow [32]. This evidence suggests that age-related changes in resident macrophages may differ between male and female mice. Given that we only studied male mice, further investigations using female mice are needed.

There are several limitations in the present study. First, only male mice were used. Second, we did not separate NP and AF tissues for analysis. Third, how a reduction in resident macrophages is associated with IVD degeneration remains unclear. Finally, resident macrophages comprise a heterogeneous population. However, the roles of these individual populations remain unclear.

## 5. Conclusions

Resident macrophages decreased with age in IVDs, which may be associated with the concomitant decrease in TGF-*β*. Our findings provide new insights into the mechanisms of age-related IVD pathology.

## Figures and Tables

**Figure 1:** Flow cytometry analysis of the macrophage population in intervertebral discs of young and aged mice. Dot plots showing CD11b+ and CD11b+ CD206+ cells in intervertebral discs (IVDs) of (a) young (age 4 months) and (b) aged (age 18 months) mice. The *x*-axis indicates CD206 and the *y*-axis indicates CD11b. (c) Percentage of CD45+ CD11b+ cells in IVDs (*n* = 5). (d) Percentage of CD11b+ CD206+ cells in IVDs (*n* = 5). ^∗^*P* < 0.05 compared with young mice.

**Figure 2:** Expression of *CD11b*, *Cd206*, and *Tgfb* in intervertebral discs of young and aged mice. Expression of (a) *Cd11b*, (b) *Cd206*, and (c) *Tgfb* in intervertebral discs of young (age 4 months) and aged (age 18 months) mice. ^∗^*P* < 0.05.

**Figure 3:** Effect of TGF-*β* on M2 marker expression in vitro. Disc macrophages derived from young (age 4 months) and aged (age 18 months) mice were stimulated with *α*-MEM (control), 10 ng/ml mouse recombinant (mr) TGF-*β*+10 ng/ml IL-10 (TGF/IL10), or 10 ng/ml mrTGF-*β* +10 ng/ml IL-10 +10 *μ*M SB431542 (TGF/IL10/SB431542) for 24 h (*n* = 5). Relative expression was determined based on expression in control samples. ^∗^*P* < 0.05 compared to vehicle.

**Figure 4:** Effect of a TGF-*β* inhibitor on *Cd206* expression in vivo. *Cd206* expression following administration of vehicle (DMSO) and TGF-*β* inhibitor (SB431542) to (a) young and (b) aged mice (*n* = 10 for each group). ^∗^*P* < 0.05 compared to vehicle.

## Data Availability

The data used to support the findings of this study are available from the corresponding author upon request.
